# Bioassay's Directed Isolation-Structure Elucidation and Molecular Docking of Triterpenes from *Persea duthiei* against Biologically Important Microbial Proteins

**DOI:** 10.1155/2022/3839271

**Published:** 2022-05-27

**Authors:** Najeeb Ullah, Shan Zeb, Fozia, Shah Rukh, Shafiullah Khan, Ijaz Ahmad, Shakeel Ahmad, Nisar Ahmad, Amal Alotaibi, Riaz Ullah

**Affiliations:** ^1^Department of Biochemistry, Bahauddin Zakariya University, Multan, Punjab, Pakistan; ^2^Department of Chemistry, Kohat University of Science & Technology, Kohat, KPK, Pakistan; ^3^Biochemistry Department, Khyber Medical University Institute of Medical Sciences, Kohat, KPK, Pakistan; ^4^Department of Pharmacy, Abasyn University, Ring Road, Peshawar 25120, KPK, Pakistan; ^5^Department of Botanical & Environmental Sciences, Kohat University of Science & Technology, Kohat 26000, KPK, Pakistan; ^6^Department of Basic Science, College of Medicine, Princess Nourah Bint Abdulrahman University, P.O. Box 84428, Riyadh 11671, Saudi Arabia; ^7^Department of Pharmacognosy (MAPPRC), College of Pharmacy, King Saud University, Riyadh, Saudi Arabia

## Abstract

The research work presented in this study is mainly concerned with the bioactivity-directed phytochemical and biological evaluation of *Persea duthiei*. *Persea duthiei* is a typical medicinal plant used to treat a variety of ailments such as asthma, edema, and bronchitis. Ethyl acetate, n-hexane, n-butanol, and compounds that are soluble in water were used to examine the antibacterial as well as antifungal capacities of the plant. The antibacterial activity of the soluble parts of ethyl acetate and n-hexane against *Escherichia coli, Staphylococcus aureus, Salmonella typhi,* and *Bacillus subtilis* was high, even though there was no activity against *Pseudomonas aeruginosa*. Likewise, the n-hexane and ethyl acetate fractions were found to have substantial efficacy against several fungal strains such as *Aspergillus flavus, Aspergillus fumigates, Fusarium solani,* and *Aspergillus niger,* but not against *Candida glabrata*. Among the studied fractions, the ethyl acetate soluble fraction had potent antibacterial activity against all of the tested species. This fraction was submitted to phytochemical analysis utilizing various chromatographic methods for the extraction of various pure components. As a consequence, four compounds were isolated, and their structures were elucidated using various spectroscopic methods such as IR, EIMS, HR-EIMS, ^1^H-NMR, ^13^C-NMR, NOESY, COSY, HMBC, and HMQC. Urs-12-en-3*β*-ol (*α*-amyrine) **(**1**),** Urs-12-ene-2*α*-3*β*-diol (chamaedrydiol) **(**2**),** 3*β*-hydroxyurs-12-en-28-aldehyde (ursolic aldehyde) **(**3**),** and 12-oleanex-3*β*-ol (*β*-amyrine) **(**4**)** were extracted. Compounds 1, 2, 3, and 4 were examined for antibacterial and antifungal activity and found to have zones of inhibition ranging from 0 to 11 mm against tested bacteria strains and percent inhibition ranging from 0 to 25 percent against fungus strains. Compounds 1 and 4 showed strong efficacy against the investigated fungal species, with a 25% inhibition rate. In the case of antibacterial activity, compounds 4 and 1 showed potent activity with zones of inhibition of 11 mm and 10 mm, respectively. Compounds 2 and 3 were observed to have nonsignificant antimicrobial activity. However, docking studies reflected the complex formation of compound 1 with beta-hydroxyacyl-ACP dehydratase HadAB and *S. aureus* tyrosyl-tRNA synthetase and compound 2 with topoisomerase II DNA gyrase complex, and they were reported to have antibacterial properties. Similarly, compound 4 was discovered to be well compatible with the lanosterol 14-demethylase (fungal enzyme) and is thus regarded as having antifungal capabilities. Chimera software was used to identify the binding pockets of these complexes. These results indicated that *Persea duthiei* is a valuable source of medicinal compounds for medication development.

## 1. Introduction

Humans as well as other living organisms are the victims of disease-causing microorganisms (including bacteria and viruses). Besides being disease-causing agents, these microorganisms are gaining resistance against antibiotics as diagnosed in many hospitals throughout the world [1]. With the increase in gaining multidrug resistance among microorganisms, the discovery of broad-spectrum antibiotics with modified and improved activity is gaining more interest in order to overcome diseases. Nature is a gift for us that is rich in antimicrobial ingredients; among them plants are rich in medicinal ingredients. The application of plants as a source of effective medicine is an urge throughout the world [2]. Medicinal plants are used to treat a variety of disorders mainly due to their low cost and high efficacy. However, the limited knowledge about their dosage, safety, liability, and harmful or allergic ingredients prevents doctors from prescribing them for medicinal purposes [3]. The reasons behind multiple antibiotic resistance in many microbial strains are their gene mutations, alternation in microbial structure, and excessive intake of nonspecific antibiotics for the treatment of various disorders. These modifications induce the treatment of microbial infections with the help of herbal medicines. Although a large number of medicinal plants have been examined in order to evaluate their antimicrobial properties, there is still a gap in satisfactory screening. Medicinal plants are a rich source of phytochemicals like alkaloids, flavonoids, glycosides, lactones, resins, sterols, tannins, and volatile oils, due to the natural synthesis of these bioactive compounds in plants. Phytochemicals are biologically active compounds that play a leading role in the treatment of various infections including microbial infections and inflammation [4–6]. The gain of resistance against drugs is a main issue in the identification of drugs for the therapy of microbial infections. Therefore, it is our urgent need to reduce the consumption of antibiotics by providing treatments for microbial infection with the help of novel natural drugs. This urge is fulfilled by the utilization of medicinal plants as well as their phyto-constituents as suitable antimicrobial drugs. *Persea* is a genus in the Lauraceae family that belongs to the oldest subtribe. In the Buner area of Pakistan, *Persea duthiei* is known by the local name “Gul-e-namair.” It is found mostly in Pakistan, India, and Burma and is also found across the western Himalayas [7]. Medicinal plants are used for the treatment of different infections. These plants contributed as a source of inspiration to novel therapeutic compounds as well as color, flavor, and taste of food [8, 9].

*Persea duthiei* is a medicinal plant with valuable medicine properties; the rootstocks, in particular, are bitter, acrid, hot, harsh, and vigorous. It is most commonly used to treat asthma, emphysema, bronchitis, pain, bad breath, blood problems, and vomiting [10]. The oils of *Persea duthiei's* fruits, leaves, and flowers were studied, and forty components were discovered. One of its oils, i.e., sesquiterpenoids, is present with a percentage of 84.2% in flower, 83% in fruit, and 35.7% in leaves. Other major components (36%) of leaf oil are monoterpene hydrocarbons. Sesquiterpenoids are represented by *α*-pinene (10%), limonene (10.1%), p-cymene (3.5%), *β*-pinene (10%), (E)-nerolidol (13.2%), *β*-caryophyllene (5.8%), epi-cubebol (5.8%), and *β*-eudesmol (4%). Besides epi-cubebol in flower oil, the (E)-nerolidol is also present in great quantity [11]. *Persea* genus is rich in phytochemical contents like flavonoids, terpenes, alkaloids, phytosterols (*β*-sitosterol), and essential oils [12].

The antibacterial activity of crude extract and several solvent soluble fractions derived from *Persea duthiei* is reported in this research. The plant's ethyl acetate soluble fraction was discovered to have the most antibacterial potential; thus, it was subjected to column chromatography. Four chemicals (1–4) were recovered as a result of sequential column chromatography of the ethyl acetate soluble fraction. Modern spectroscopic approaches, including 1D and 2D NMR techniques, were used to determine the structures of compounds 1–4 (Figure 1). Both physical and spectral data of compounds 1–4 agreed completely with those previously published in the literature [13–15]. Despite the fact that the structures of compounds 1–4 have been disclosed previously, we are presenting their antibacterial activity and docking investigations against key microbial proteins for the first time.

## 2. Materials and Methods

### 2.1. Collection of Plant

A plant taxonomist, Professor Mehboob Ur Rehman, in the Plant Sciences Section of Postgraduate Jahanzeb College, Saidu Sharif, Swat, Pakistan, collected the plant *Persea duthiei* and identified it with a specimen voucher number HPGJC 127 lodged there.

### 2.2. Extraction and Fractionation

The entire plant *Persea duthiei* was collected, dried in shade with the presence of air, sliced, and powdered to a coarse (fine) consistency. At room temperature, the powdered plant, weighing six kg, was extracted three times with methanol (MeOH). This methanolic extract was then evaporated in rotary evaporator under low pressure, yielding dark green thick (like syrup) residue; dried; and weighed. It weighed around 711 grams. Then, this residue was partitioned into different sections with the help of a separating funnel. This methanolic extract was subsequently divided into solvents with varying polarity, such as n-hexane, n-butanol, EtOAc, and water soluble fractions. The antibacterial activity of the crude extract and subsequent soluble fractions was tested, with the ethyl acetate fraction proving to be the most effective.

### 2.3. Isolation of Pure Compounds

The extract's ethyl acetate fraction (eighty-six grams) was subjected to column chromatography. For the process of elution, different solvents having different polarities were used. Elution was performed using the solvents having a gradient of increasing polarity, with the sequence of ascending polarity being (n-hexane)⟶(n-hexane-ethyl acetate)⟶(pure ethyl acetate)⟶(ethyl acetate-methanol) and the final elution being pure methanol.

After that, the eluted fractions with identical TLC characteristics were blended together. As a result of the compilation procedure, four (04) subfractions were obtained: F1, F2, F3, and F4. These four (04) subfractions were then submitted to repeated column chromatography for further purification. Fraction F1 was rechromatographed after being eluted with n-hexane-ethyl acetate (8 : 2). One pure chemical was obtained from fraction F1 [13]. Elution in the (6 : 4) fraction of n-hexane-ethyl acetate yielded fraction F2, which was then subjected to column chromatography. This fraction produced two compounds, 2 [11] and 3 [16], on successive chromatography eluted with two different ratios of n-hexane-ethyl acetate (9 : 1 and 1.5 : 8.5), respectively. Fraction F4 was separated and then subjected to column chromatography after being eluted with n-hexane-ethyl acetate in a ratio of 3 : 7. One pure chemical, 4 [13], was also obtained from this fraction, which was eluted using n-hexane-ethyl acetate (4 : 6).

### 2.4. Bioscreening

To assess their antimicrobial potential, soluble fractions of different solvents and their components extracted, 1 to 4, from *Persea duthiei* were tested for their antibacterial and antifungal activity.

#### 2.4.1. Microbial Strains

The fractions of *Persea duthiei* in different solvents (ethyl acetate, methanol, n-butanol, and n-hexane) and the pure compounds 1–4 were tested against ten microbial species. *Bacillus subtilis, Escherichia coli, Pseudomonas aeruginosa, Salmonella typhi,* and *Staphylococcus aureus* are the five bacterial pathogens, while *Aspergillus flavus, Aspergillus fumigates, Aspergillus niger, Candida glabrata*, and *Fusarium solani* are the five fungal pathogens. The microbes were taken from Dr. Panjwani Center for Molecular Medicine and Drug Research at the University of Karachi in Pakistan (ICCBS).

#### 2.4.2. Antibacterial Assay

Various strains of bacterial species were subcultured in order to create a freshly cultured bacterial species for the evaluation of antibacterial activity. As a result, each colony from a different bacterial strain was injected into the nutrient broth and cultivated for one day at room temperature (37°C). The dissolved 19 g nutritious agar medium in 1 L distilled water was then autoclaved at 121°C for half an hour. After chilling, the media were put onto 14 cm Petri plates to make 75 mL of solid media. In these solid media, 7 holes were drilled with a sterile cork borer (8 mm). To evaluate the antibacterial activity of various fractions, the agar diffusion method was used. Each bacterial strain was inoculated in its own Petri dish. To make the stock solution, 15 mg per mL of each part was combined with DMSO (dimethyl sulfoxide). In such precise holes, 100 L solution of each fraction, DMSO solution as a negative control, and doxycycline as as a positive control were employed. The bacterial cultures along with solvent soluble fractions were cultivated for 24 hours at 37 degrees Celsius. According to the prior protocol [17], the zone of each hole was measured in millimeters.

#### 2.4.3. Antifungal Assay

To obtain fresh cultures for each species, the old fungal strains were subcultured. For cultivating fungal strains, nutrient broth medium was utilized, and the resultant cultures were cultured at 280°C for 7 days. The disc diffusion method was employed to assess antifungal activity in different solvent soluble fractions of this plant. Through point inoculation, the fungal strains were injected on distinct agar media, namely, Potato Dextrose Agar (PDA) plates. The experiment next employed 100 microL of the store solution (12 mg from each fraction dissolved in 2 ml of DMSO); pure DMSO as a negative control; and 12 mg/mL antibiotic, i.e., miconazole, as a positive control. The activity of each strain was assessed after 7-day (280°C) incubation [17].

### 2.5. Physical and Spectral Data of Compounds 1–4

#### 2.5.1. Urs-12-en-3*β*-ol (1)

Amorphous solid; M.P 188°C; IR (KBr) cm^−1^ 3512, 1638; ^1^H-NMR (CDCl_3_, 400 MHZ); □ 5.11 (1H, t, *J* = 3.6 Hz, H-12), 3.22 (1H, dd, *J* = 10.4, 7.2 Hz, H-3), 2.35 (2H, m, H-11), 1.98 (1H, m, H-9), 1.95 (2H, m, H-1), 1.89 (1H, m, H-18), 1.68 (2H, m, H-15), 1.52–1.60 (9H, m, H-19, 16, 7, 6, 2), 1.40–149 (5H, m, H-20, 21, 22), 1.11 (3H, s, CH_3_), 1.05 (3H, s, CH_3_), 0.99 (3H, s, CH_3_), 0.97 (3H, s, CH_3_), 0.89 (1H, m, H-5), 0.85 (3H, s, CH_3_), 0.83 (3H, s, CH_3_), 0.81 (3H, s, CH_3_), 0.79 (3H, s, CH_3_); ^13^C-NMR (CDCl_3_, 125 MHZ); □ 139.60 (C-13), 124.40 (C-12), 77.22 (C-3), 59.07 (C-18), 55.18 (C-5), 47.72 (C-9), 42.09 (C-14), 41.54 (C-22), 40.02 (C-8), 39.68 (C-19), 39.62 (C-20), 38.72 (C-1), 38.06 (C-4), 36.96 (C-10), 33.76 (C-17), 32.66 (C-7), 31.27 (C-21), 28.14 (C-15, 23, 28), 27.25 (C-2), 26.63 (C-16), 23.39 (C-11), 23.28 (C-27), 21.40 (C-30), 18.37 (C-6), 17.48 (C-29), 16.81 (C-26), 15.63 (C-24), 15.60 (C-25); HREI-MS: *m/z* calc for C_30_H_50_O [M]^+^ 426.386 and was found as 426.382 [13].

#### 2.5.2. Urs-12-ene-2*α*-3*β*-Diol (2)

Amorphous solid; M.P 219–220°C; IR (KBr) cm^−1^ 3510, 1635; ^1^H-NMR (CDCl_3_, 400 MHZ); □ 5.32 (1H, t, *J* = 3.8 Hz, H-12), 3.68 (1H, m, H-2), 3.01 (1H, d, *J* = 7.6H, H-3), 2.09–2.02 (5H, m, H-11, 1, 9), 1.98 (1H, m, H-18), 1.74 (2H, m, H-15), 1.63 (2H, m, H-22), 1.60–1.51 (9H, m, H-21, 6, 16, 7, 19), 1.40 (1H, m, H-20), 1.23 (3H, s, CH_3_), 1.05 (3H, s, CH_3_), 1.02 (3H, s, CH_3_), 1.00 (3H, s, CH_3_), 0.98 (3H, s, CH_3_), 0.90 (1H, m, H-5), 0.89 (3H, s, CH_3_), 0.81 (3H, s, CH_3_), 0.77 (3H, s, CH_3_); ^13^C-NMR (CDCl_3_, 125 MHZ); □ 139.60 (C-13), 124.17 (C-12), 83.98 (C-3), 69.04 (C-2), 59.03 (C-18), 55.20 (C-5), 47.66 (C-9), 42.13 (C-14), 41.50 (C-1, 22), 40.07 (C-8), 39.64 (C-19), 39.58 (C-20), 38.34 (C-4), 37.12 (C-10), 33.37 (C-17), 32.82 (C-7), 31.23 (C-21), 28.39 (C-23, 28), 28.06 (C-16), 26.55 (C-15), 23.42 (C-11), 23.26 (C-27), 21.41 (C-30), 18.33 (C-6), 17.46 (C-29), 16.97 (C-26), 16.89 (C-25), 16.78 (C-24); HREI-MS: *m/z* calc for C_30_H_50_O_2_ [M]^+^ 442.381 and was found as 442.377 [14].

#### 2.5.3. 3*β*-Hydroxyurs-12-en-28-Aldehyde (3)

Yellowish amorphous solid; M.P 219–220°C; IR (KBr) cm^−1^ 3516, 3511, 1696; ^1^H-NMR (CDCl_3_, 400 MHZ); □ 9.20 (1H, s, CHO), 5.30 (1H, t, *J* = 3.6 Hz, H-12), 3.12 (1H, dd, *J* = 7.6, 4.8 Hz, H-3), 2.61 (2H, m, H-22), 2.31–2.30 (3H, m, H-11,9), 1.97 (3H, m, H-1, 18), 1.86–1.80 (4H, m, H-21,2), 1.65 (2H, m, H-15), 1.58–1.49 (8H, m, H-6, 16, 7, 19, 20), 1.11 (3H, s, CH_3_), 1.06 (3H, s, CH_3_), 0.96 (3H, s, CH_3_), 0.94 (3H, s, CH_3_), 0.90 (3H, s, CH_3_), 0.88 (3H, s, CH_3_), 0.84 (1H, m, H-5), 0.75(3H, s, CH_3_); ^13^C-NMR (CDCl_3_, 125 MHZ); □ 207.56 (C-28), 137.80 (C-13), 123.26 (C-12), 77.22 (C-3), 55.21 (C-5), 55.21 (C-18), 52.63 (C-17), 47.57 (C-9), 42.18 (C-14), 40.42 (C-8), 38.99 (C-19), 38.70 (C-1), 38.62 (C-20), 38.50 (C-4), 36.95 (C-10), 32.75 (C-7), 31.88 (C-21), 30.19 (C-22), 25.50 (C-23), 27.75 (C-2,15), 26.75 (C-16), 23.31 (C-11,27), 21.08 (C-30), 18.31 (C-6), 17.22 (C-24,26), 16.66 (C-29), 15.62 (C-25); HREI-MS: *m/z* calc for C_30_H_48_O [M]^+^ 440.365 and was found as 440.361 [15].

#### 2.5.4. 12-Oleanex-3*β*-ol (4)

Solid; IR (KBr) cm^−1^ 3510, 1636; ^1^H-NMR (CDCl_3_, 400 MHZ); □ 5.11 (1H, t, *J* = 3.6 Hz, H-12), 3.21 (1H, dd, *J* = 12, 4 Hz, H-3), 2.33 (2H, m, H-11), 2.28 (1H, m, H-9), 1.98 (1H, m, H-18), 1.94 (2H, m, H-1), 1.68 (2H, m, H-15), 1.65 (2H, m, H-2), 1.57–151 (8H, m, H-6,16,7,19), 1.48–142 (4H, m, H-21,22), 1.20 (3H, s, CH_3_), 1.12 (3H, s, CH_3_), 1.11 (3H, s, CH_3_), 0.96 (3H, s, CH_3_), 0.90 (3H, s, CH_3_), 0.89 (3H, s, CH_3_), 0.85 (3H, s, CH_3_), 0.82 (1H, m, H-5), 0.76 (3H, s, CH_3_); ^13^C-NMR (CDCl_3_, 125 MHZ); □ 145.30 (C-13), 122.68 (C-12), 79.04 (C-3), 55.22 (C-5), 47.63 (C-9,18), 45.89 (C-19), 41.12 (C-14), 39.27 (C-4,8), 38.42 (C-1,22), 37.08 (C-10), 33.80 (C-21), 32.66 (C-7), 32.21 (C-17), 30.18 (C-20), 33.06 (C-30), 28.11 (C-28), 27.69 (C-16), 27.19 (C-2,15), 25.91 (C-23), 23.41 (C-11), 23.28 (C-27), 23.57 (C-29), 18.32 (C-6), 17.06 (C-26), 15.56 (C-25), 15.33 (C-24); HREI-MS: m/z calc for C_30_H_50_O [M]^+^ 426.386 and was found as 426.382 [13].

### 2.6. Docking Study

Molecular docking facilitates the comparison of potential binding interactions of identified chemical compounds with targeted proteins. The three-dimensional or 3D shape of targeted proteins (*S. aureus*. tyrosyl-tRNA synthetase, topoisomerase II DNA gyrase, beta-hydroxyacyl-ACP dehydratase HadAB, and lanosterol 14-demethylase enzyme with PDB codes 1JIJ, 2XCT, 4RLT, and 4WMZ) was obtained from RCSB PDB [18]. ChemDraw Professional v17 was used to sketch the ligand molecules [19]. The structures of receptors were generated with the help of the MakeReceptor Wizard module of the OpenEye Scientific Software, and the ligands' correct conformers were prepared with the help of the OMEGA module of the same software [20]. The structures of receptors and conformers of ligands were required before performing the protocol of molecular docking in the FRED ligand docking module. This software demands input conformers for each targeted compound. For that purpose, the ligands' conformers were developed with the help of OMEGA 3.0.0 [21]. For the generation of multiple conformers, the default setting of OMEGA was utilized. For the generation of grids of receptors the Pdb2Receptor grid generation module was used. The grids were tailored to each individual protein. For example, the grid against the *S. aureus* gyrase complex was developed around ciprofloxacin, but the grid against the *S. aureus* tyrosyl-tRNA synthetase complex was built around co-crystal SB-239629 ligand. Additionally, against co-crystallized *S. cerevisiae* and beta-hydroxyacyl-ACP dehydratase HadAB, the grid was formed around co-crystallized fluconazole ligand and fisetin. Boundary box for each targeted protein was spacious enough to cover the overall binding region, and it was obtained by setting it at the default value. The docking process was optimized by re-docking between the active sites of the targeted protein and the co-crystal ligand. The FRED module constructed different poses for each targeted ligand, and the pose with the lowest chemguass4 value was chosen for further analysis. The Discovery Studio client v16.1.0 was used to analyze the optimal docked binding relationship [22].

## 3. Results and Discussion

The methanolic extract prepared from *Persea duthiei* plant was partitioned into n-hexane, ethyl acetate, n-butanol, and water-soluble portions to isolate the physiologically essential parts. As a result, four terpenoids with structures similar to those indicated in Figure 1 were revealed. The antibacterial and antifungal properties were tested on the soluble fractions as well as the separated pure components.

### 3.1. Antibacterial Activity of Fractions

The antibacterial activity of *Persea duthiei* extract is shown in Table 1. *Persea duthiei* was tested for antibacterial efficacy against five different bacteria strains (*E. coli, B. subtilis, P. aeruginosa, S. typhi,* and *S. aureus*). With the exception of *P. aeruginosa*, all studied microorganisms showed significant efficiency in relation to the ethyl acetate and n-hexane fractions (Table 1). The ethyl acetate fraction inhibited *E. coli, B. subtilis*, *P. aeruginosa, S. typhi,* and *S. aureus* in zones of 8 mm, 3 mm, 16 mm, 9 mm, and 12 mm, respectively. However, against *E. coli, B. subtilis*, *P. aeruginosa, S. typhi,* and *S. aureus*, the percentage of n-hexane had the zones of inhibition of 11 mm, 2 mm, 7 mm, 10 mm, and 8 mm. Because the inhibition zone for the n-butanol and the aqueous fraction is so much smaller, they have less antibacterial activity.

### 3.2. Antifungal Activity of Fractions

Table 2 shows the antifungal activity of *Persea duthiei's* various solvent soluble separated fractions. All of the fungus strains examined demonstrated strong activity against the ethyl acetate and n-hexane fractions. It is also clear from Table 2 that each fungal strain shows 100 percent growth against aqueous fractions of *Persea duthiei*. However, the butanol fractions showed antifungal activity against only two strains (*A. flavus* and *F. solani*).

### 3.3. Structural Elucidation of Compounds 1–4 Isolated from *Persea duthiei*

The ethyl acetate soluble fraction was submitted to column chromatography since it showed the maximum activity of all the fractions examined, giving four chemicals (1–4).

#### 3.3.1. Urs-12-en-3*β*-ol (*α*-Amyrine) (1)

Compound 1 was synthesized in powder form with amorphous nature and melted at 188°C. The compound's chemical formula was determined as C_30_H_50_O using HR-EIMS with a molecular peak ion at m/z 426. Compound 1 in its IR spectra indicated a hydroxyl group maximum absorption at 3512 cm^−1^ and a carbon-carbon double bond absorption peak at 1638 cm^−1^. Both ^13^C- and ^1^H-NMR spectra were found to be very similar to those reported for compound 1 [13] and are provided in the experimental section of the article.

#### 3.3.2. Urs-12-ene-2*α*-3*β*-Diol (Chamaedrydiol) (2)

This compound was synthesized as an amorphous solid using an n-hexane–ethyl acetate (6 : 4) solvent system and a melting point of 219–2200°C. HR-EIMS and ^13^C-NMR (DEPT, BB) confirmed compound 2's molecular formula as C31H52O2, with a peak of molecular ion at m/z 456. In the IR spectra, OH group presented its absorption bands at 3510 cm^−1^, while a double bond (C=C) had absorption bands at 1635 cm^−1^. The physical and other spectrum data above validated the structure of compound 2 as Urs-12-ene-2-3-diol (chamaedrydiol), which agrees with those reported in the literature [13] and is also included in the experimental portion of the paper [12].

#### 3.3.3. 3*β*-Hydroxyurs-12-en-28-Aldehyde (Ursolic Aldehyde) (3)

Through column chromatography, an amorphous solid of yellow color material, i.e., compound 3, was recovered from F4 fraction using an n-hexane to ethyl acetate ratio of 7 : 3. When compound 3 was exposed to the iodine chamber, it appeared as a yellow spot. The provided compound's IR spectra reflected the absorption for the OH at 3511 cm^−1^, for the carbonyl group at 1696 cm^−1^, and for the C=C olefinic at 3516 cm^−1^. HR-EIMS technology revealed a peak for molecular ion at m/z 440.00, confirming the chemical formula C30H48O2 (calc for C30H48O2, 440.00). The ^13^C-NMR and ^1^H-NMR spectrum data for compound 3 [15, 23] were found to be extremely similar to those available in literature and are included in the experimental portion of the paper.

#### 3.3.4. 12-Oleanex-3*β*-ol (*β*-Amyrine) (4)

After washing with methanol, the amorphous solid of compound 4, i.e., *β*-amyrine, was isolated in the ethyl acetate soluble fraction of *Persea duthiei*'s MeOH extract and crystallized to a colorless needle-like crystal. HR-EIMS was used to detect a molecular ion peak at m/z 426.38, which corresponded to the C_30_H_50_O as its chemical formula. Infrared spectra represent absorption peaks for the OH group at 3510 cm^−1^ and a trisubstituted double bond at 1636 cm^−1^. Compound 4's ^1^H-NMR spectra and ^13^C-NMR assignment were indistinguishable from those described in the literature for *β*-amyrine [13], which is also supplied in the article's experimental section.

### 3.4. Bio-screening of Compounds

Antibacterial and antifungal properties were tested on the four identified compounds, 1–4, at a concentration of 28 g/ml. Compound 4 was shown to be more active than compounds 2 and 3, whereas compound 1 had the second highest level of antibacterial activity for all the targeted bacterial strains with the exception of *B. subtilis* as mentioned in Table 3. Compounds 4 and 1 showed antibacterial activity for the investigated bacterial strains. However, in terms of antifungal activity, compound 1 demonstrated the most activity against all fungal strains, followed by compound 4.  Table 4 shows that compounds 2 and 3 have no substantial action.

### 3.5. Structure-Activity Relationship of Isolated Compounds

The antimicrobial activities of all the four isolated compounds were examined by evaluating the structure-activity relationship of these compounds.

Compound 1 **(**i.e., *α*-amyrine), a pentacyclic triterpene, is a pharmacological important compound that exhibits antimicrobial and anti-inflammatory as well as anticancer properties [16, 24]. Compound 1 (*α*-amyrine) shows more antimicrobial activity against each targeted microbial strain. The reason behind the pharmacological importance of *α*-amyrine is represented by evaluating the structure-activity relationship of compound 1. The presence of OH group at R2 is involved in the formation of H-bonding with the membrane proteins of bacteria, ultimately leading to lysis or rupture of microbial cell [25] that is represented in their zone of inhibition for bacterial strains (Table 3) and percent inhibition for fungal strains (Table 4). Compound 2 (i.e., chamaedrydiol) has minimum antimicrobial activities compared to the other 3 compounds. The reason behind this least activity is exhibited in its structure. It has two adjacent OH groups at R1 and R2 positions; these adjacent OH groups generally reduce the strength of H-bonding, thereby resulting in the least activity against bacteria and fungi [26]. Compound 3 (i.e., ursolic aldehyde) has the least antibacterial activity against three strains of bacteria (*S. typhi, P. aeruginosa,* and *S. aureus)* and has near to zero antibacterial activity against *E. coli* and *B. subtilis*. This low or no activity of (ursolic aldehyde) is based on the presence of carbonyl group (C=O) at the R3 position. This carbonyl group hinders the antimicrobial activity of compounds [23, 27]. However, the presence of the OH group at R2 is involved in the formation of H-bond with microbial membrane protein, so this compound has weak antimicrobial activity [27]. Compound 4, (i.e., *β*-amyrine) is also a pentacyclic triterpene; its pharmacological as well as antibacterial activities are similar to those of compound 1. The antibacterial activities of both compounds are also relatable to each other [24, 25].

### 3.6. Molecular Docking Studies

The predicted binding relationship of ligands with physiologically significant targeted proteins is evaluated using molecular docking. Each isolated chemical was subjected to docking studies to identify its directing of binding inside the pockets at the active site of the target proteins. HadAB, *S. aureus* tyrosyl-tRNA synthetase, and topoisomerase II DNA gyrase, along with one fungus protein, lanosterol 14-demethylase (CYP51), were examined to determine whether they may be exploited as therapeutic targets for antibacterial and antifungal drug development. Tables 5–8 show the binding affinity of all compounds under investigation against 3 bacterial and one fungal proteins using the FRD docking program's chemguass4 score. FRED uses multi-conformer docking techniques, which entail generating a number of conformers with low energy one at a time and firmly docking each one.

Bacterial beta-hydroxyacyl-ACP dehydratase HadAB is an enzyme that is involved in catalyzing the dehydration step of bacterial fatty acid elongation [28]. The formation of complex having this enzyme with the targeted compounds can inhibit the significant role of this dehydratase enzyme ultimately leading to antibacterial therapy. By putative binding of four isolated compounds with this enzyme in docking studies, the FRED score of all compounds is obtained and represented in Table 5. The values of the FRED score indicate that compound 1 has a more putative binding with this enzyme, having −11.85 FRED score. Structure-activity relationship also represents the comparatively more antibacterial activity of compound 1 against bacterial strains. The docking results suggest that the hydroxyl group as well as the hydrophobic portion of these compounds is interfering with the microbial proteins through various intermolecular interactions. Further, crystallographic studies can confirm the part of the compound interacting with the proteins.

Figure 2 depicts the synthesis of compound 1 in association with beta-hydroxyacyl-ACP dehydratase HadAB.

In docking study, three parameters were assessed: the binding affinity expressed in kcal/mol, the bonding interactions between the amino acid residues of the target protein and the atoms of the ligand, and the bond distance of these interactions, as shown in Table 9.

*S. aureus* tyrosyl-tRNA synthetase is a bacterial enzyme, catalyzing the activation of tyrosine and its transfer to tRNA during translation of various important bacterial proteins [29]. The putative binding of four isolated compounds with this enzyme is evaluated in FRD docking software. FRED scores of all compounds are obtained and represented in Table 7. The values of FRED score indicate that compound 1 has a more putative binding affinity with this enzyme, with a FRED score of −8.23. Compound 1 has a higher antibacterial activity than compound 2 against the bacterial strains, as shown by the structure-activity relationship.

The formation of compound 1–*S. aureus* tyrosyl-tRNA synthetase complex is represented in Figure 3. Three parameters were evaluated using docking analysis: first is the binding affinity expressed in kcal/mol, second is the interactions between the amino acid residues of the target protein and the atoms of ligand, and third is the bond distance of these interactions as represented in Table 10.

Topoisomerase II DNA gyrase is a bacterial enzyme that is involved in introducing turns in DNA (i.e., negative superhelical turns), so it is involved in the replication of bacterial strains [31]. However, the formation of a complex having bioactive compounds with this enzyme can retard the normal replication of microbes. The putative binding of four isolated compounds with this enzyme was evaluated with FRD docking software. FRED scores of all compounds are obtained and represented in Table 7. The values of FRED score show that compound 2 has more putative binding with this enzyme, with a FRED score of −1.48.

The formation of compound 2–topoisomerase II DNA gyrase complex is represented in Figure 4. Three parameters were evaluated using docking analysis: first is the binding affinity expressed in kcal/mol, second is the bonding interactions between the amino acid residues of the target protein and the atoms of ligand, and third is the bond distance of these interactions as shown in Table 11.

Lanosterol 14*α*-demethylase is a fungal enzyme, involved in the synthesis of a necessary component (ergosterol) of the cell membrane in fungi [33]. Inhibition of this enzyme leads to reduction of ergosterol in fungal cell membrane and formation of toxic metabolites [34]. Both these effects are fungistatic for many pathogenic fungi. For the synthesis of novel antifungal medications, this enzyme has gained much importance. Docking studies revealed that compound 4 showed more stable complex with this enzyme, with chemguass4 score of −12.89, than the other three compounds (Table 8).

The formation of compound 4–lanosterol 14*α*-demethylase complex is represented in Figure 5. Three parameters were evaluated using docking analysis: first is the binding affinity expressed in kcal/mol, second is the interactions between the amino acid residues of the target protein and the atoms of ligand, and third is the bond distance of these interactions as listed in Table 12.

The docking results between the enzymes *β-*hydroxyacyl-ACP dehydratase (PDB ID: 4rlt) and tyrosyl-tRNA synthetase (PDB ID: 1jij) with compound 1 are visualized in 3 dimensions and shown in Figure 6. Similarly, the binding pocket visualization and active site residue interaction of topoisomerase II DNA gyrase (PDB ID: 2xct) with chamaedrydiol and lanosterol 14*α*-demethylase enzyme (PDB ID: 4wmz) with compound 4 are shown in Figure 7. The 3D visualizations were performed by Chimera software [35].

## 4. Conclusion

The findings of this article concluded that *Persea duthiei* showed potent antibacterial and antifungal properties due to having bioactive ingredients (phytochemicals). Among different solvent soluble fractions, ethyl acetate and n-hexane fractions exhibited decent antimicrobial potency. Ethyl acetate soluble fraction yielded four compounds that served as antimicrobial target inhibitors/prodrugs. Compound 1 (*α*-amyrine) and compound 4 (*β*-amyrine) showed more significant antimicrobial properties due to their potential interaction with the microbial membrane proteins. Molecular docking studies also reflected the antimicrobial activities (antibacterial as well as antifungal activities) of these compounds by indicating the putative binding interaction with the bacterial enzyme (beta-hydroxyacyl dehydratase, tyrosyl-tRNA synthetase, and topoisomerase II DNA gyrase) and fungal enzyme (lanosterol 14*α*-demethylase) active sites, respectively. These findings may be helpful in modifying theses reported compounds, targeting the biologically significant proteins, and may help in the development of new and advanced broad-spectrum antibiotics. Further, the authors will crystallize and subsequently co-crystallize these important microbial proteins along with these four terpenoids to see their interactions in real natural environment, leading to *in vivo* inhibition studies.

## Figures and Tables

**Figure 1:** The structure of four isolated compounds: (a) compound 1; (b) compound 2; (c) compound 3; (d) compound 4.

**Figure 2:** Putative binding interaction of compound 1 with the bacterial enzyme HadAB. Residues of compound 1 are interacting with the enzyme active site amino acid residues like THR138 and THR140 (shown in yellow sticks) at the active site of bacterial beta-hydroxyacyl-ACP dehydratase HadAB [25] through hydrogen bond (dotted lines in green).

**Figure 3:** Putative binding interaction of compound 1 against bacterial *S. aureus* tyrosyl-tRNA synthetase. The THR75 (interacting with OH group of compound 1) and ASP177 (interacting with hydrogen atom of compound 1) residues of *S. aureus* tyrosyl-tRNA synthetase are hydrogen-bonded with OH group of compound 1, similar to its hydrogen bond formation with SB-284485 as previously reported. Similarly, HIS50 residue is also present in the active site of *S. aureus* tyrosyl-tRNA synthetase that interacts through hydrophobic bonding with the hydrophobic part of compound 1 in a similar fashion to that between SB-239629 and *S. aureus* tyrosyl-tRNA synthetase [30].

**Figure 4:** Putative binding interactions of compound 2 against bacterial topoisomerase II DNA gyrase. The ASP437 residue (shown in red) located at the active site of topoisomerase II DNA gyrase forms H-bond (dotted line in green) with OH group of compound 2, in a similar way to hydrogen bond formation between the GSK299423 inhibitor and the enzyme [32].

**Figure 5:** Putative binding interaction of compound 4 against fungal lanosterol 14*α*-demethylase enzyme. The amino acids LEU380, LEU383, and VAL311 in the hydrophobic core of the enzyme located in the active site are involved in the hydrophobic Van der Waals bonding with the hydrophobic residues of compound 4 [35].

**Figure 6:** The visualization of binding pockets of enzyme *β-*hydroxyacyl-ACP dehydratase (PDB ID: 4rlt) (a, b) and tyrosyl-tRNA synthetase (PDB ID: 1jij) (c, d) with *α*-amyrine. Compound 1 (depicted as a stick) is embedded in the binding pockets of enzymes. (a, b) Binding of compound 1 in the active site of enzyme *β-*hydroxyacyl-ACP dehydratase through active site residues GLN86 and GLN89 of *β*2 strand and THR138, THR140, and LEU142 of *β*5 strand forming hydrogen bond with the hydroxyl groups of the ligand. (c, d) Compound 1 bound to the tyrosyl-tRNA synthetase' active site residue THR75 that is involved in the formation of hydrogen bond with the OH group of compound 1.

**Figure 7:** Visualization of binding pockets. (a, b) The interaction between compound 2 and topoisomerase II DNA gyrase (PDB ID: 2xct) enzyme is depicted. Compound 2 (shown in yellow sticks) is involved in the formation of hydrogen bond with the DNA (red and gray) and also interacts with the ASP437 residue of this enzyme. (c, d) Docked complex of lanosterol 14*α*-demethylase enzyme (PDB ID: 4wmz) with compound 4 is depicted. This enzyme has a hydrophobic pocket (lined with VAL, LEU, PHE, and TYR), and interestingly the PHE and TYR form a hydrophobic tunnel (residues shown in red sticks) that may facilitate the stabilization and subsequent co-crystallization through the hydrophobic core of compound 4.

**Table 1:** Zones of inhibition in millimeters showing antibacterial activities of isolated fractions of *Persea duthiei* against different bacterial strains (15 mg/ml).

S. No.	Fractions	*E. coli*	*P. aeruginosa*	*S. typhi*	*B. subtilis*	*S. aureus*
1	n-Hexane	11	2	7	10	8
2	Ethyl acetate	8	3	16	9	12
3	n-Butanol	1	4	3	2	5
4	Aqueous	3	1	5	2	3
5	Doxycycline	16	19	24	22	20

**Table 2:** Antifungal activity (% inhibition) of different fractions (15 mg/ml) [17] isolated from *Persea duthiei* against five fungi strains.

S. No.	Fractions	*A. flavus*	*A. fumigates*	*A. niger*	*F. solani*	*C. glabrata*
1	n-Hexane	+, +	+	+, +	+	+
2	Ethyl acetate	+, +	+	+, +	+, +	+
3	n-Butanol	+	−	−	+	−
4	Aqueous	−	−	−	−	−
5	Miconazole	+, +, +, +	+, +, +, +	+, +, +, +	+, +, +, +	+, +, +, +

Note. (−) 100% growth; (+) 75% growth; (+, +) 50% growth; (+, +, +) 25% growth; (+, +, +, +) no growth.

**Table 3:** Zones of inhibition in millimeters showing antibacterial activities of isolated compounds 1–4 (28 *μ*g/ml) of *Persea duthiei* against different bacterial strains.

S. No.	Compounds	*E. coli*	*P. aeruginosa*	*S. typhi*	*B. subtilis*	*S. aureus*
1	Compound 1	7	8	10	1	2
2	Compound 2	8	5	0	0	3
3	Compound 3	0	5	2	0	7
4	Compound 4	9	11	9	1	5
5	Levofloxacin	16	19	24	22	20

**Table 4:** Antifungal activity (% inhibition) of compounds 1–4 (28 *μ*g/ml) isolated from *Persea duthiei* against five fungi strains.

S. No.	Compounds	*A. flavus*	*A. fumigates*	*A. niger*	*F. solani*	*C. glabrata*
1	Compound 1	+	+	+	+	+
2	Compound 2	+	−	−	−	−
3	Compound 3	−	+	−	−	−
4	Compound 4	+	+	−	+	−
5	Clotrimazole	+, +, +, +	+, +, +, +	+, +, +, +	+, +, +, +	+, +, +

Note. (−) 100% growth; (+) 75% growth; (+, +) 50% growth; (+, +, +) 25% growth; (+, +, +, +) no growth.

**Table 5:** FRED chemguass4 score of compounds 1–4 and co-crystalized reported ligand against docking with bacterial enzyme beta-hydroxyacyl-ACP dehydratase HadAB (PDB ID: 4rlt).

Compound code	FRED chemguass4 score
Compd_1	−11.85
Compd_2	−10.34
Compd_3	−11.07
Compd_4	−10.55
4RLT_cc	−14.85

**Table 6:** FRED chemguass4 score of compounds 1–4 and co-crystalized ligand against docking in bacterial enzyme *S. aureus* tyrosyl-tRNA synthetase (PDB ID: 1jij).

Compound code	FRED chemguass4 score
Compd_1	−8.23
Compd_2	−6.90
Compd_3	−7.89
Compd_4	−7.02
Co-crystalized ligand	−14.64

**Table 7:** FRED chemguass4 score of compounds 1–4 and co-crystalized ligand against docking in bacterial enzyme topoisomerase II DNA gyrase (PDB ID: 2xct).

Compound code	FRED chemguass4 score
Compd_1	−1.33
Compd_2	−1.48
Compd_3	−0.72
Compd_4	−0.99
Co-crystalized ligand	−3.25

**Table 8:** FRED chemguass4 score of compounds 1–4 and co-crystallized ligand against docking with fungal enzyme, i.e., Lanosterol 14*α*-demethylase enzyme (PDB ID: 4wmz).

Compound code	FRED chemguass4 score
Compd_1	−12.62
Compd_2	−12.72
Compd_3	−12.44
Compd_4	−12.89
Co-crystalized ligand	−11.25

**Table 9:** Molecular docking analysis of compound 1 against bacterial enzyme beta-hydroxyacyl-ACP dehydratase HadAB (PDB ID: 4rlt) on the basis of the type of bonds, the bond distances, and the interacting amino acids.

Bond type	Bond distance (Å)	Interacting amino acid of target
Hydrogen bond	2.71	A:THR140:OG1
Hydrogen bond	2.94	A:THR138:OG1
Hydrogen bond	2.71	A:THR140:OG1
Hydrogen bond	2.94	A:THR138:OG1
Hydrogen bond	2.71	A:THR140:OG1
Hydrogen bond	2.94	A:THR138:OG1
Hydrophobic	4.64	A:ILE84
Hydrophobic	4.82	A:LEU142
Hydrophobic	5.49	A:LEU142
Hydrophobic	5.24	B:MET60
Hydrophobic	5.45	A:LEU142
Hydrophobic	5.26	A:ILE84
Hydrophobic	4.58	A:LEU142
Hydrophobic	5.18	A:LEU142
Hydrophobic	3.71	A:CYS61
Hydrophobic	4.79	A:CYS61
Hydrophobic	5.03	A:TYR65
Hydrophobic	5.13	A:TYR65
Hydrophobic	5.06	A:TYR65
Hydrophobic	5.41	A:PHE72

**Table 10:** Molecular docking analysis of compound 1 against bacterial enzyme *S. aureus* tyrosyl-tRNA synthetase (PDB ID: 1jij) based on the type of bonds, bond distances, and interacting amino acids.

Bond type	Bone distance (Å)	Interacting amino acid of target
Hydrogen bond	1.84	A:THR75:OG1
Hydrogen bond	3.04	A:ASP177:OD1
Hydrogen bond	1.84	A:THR75:OG1
Hydrogen bond	3.04	A:ASP177:OD1
Hydrophobic	3.55	A:ALA39
Hydrophobic	4.17	A:ALA39
Hydrophobic	4.83	A:PRO53
Hydrophobic	4.28	A:CYS37
Hydrophobic	3.55	A:LEU70
Hydrophobic	4.84	A:TYR36
Hydrophobic	5.19	A:HIS47
Hydrophobic	4.44	A:HIS50
Hydrophobic	3.48	A:HIS50
Hydrophobic	5.14	A:TYR170

**Table 11:** Molecular docking analysis of compound 2 against bacterial enzyme topoisomerase II DNA gyrase (PDB ID: 2xct) on the basis of the type of bonds, bond distances, and interacting amino acids.

Bond type	Bond distance (Å)	Interacting amino acid of target
Hydrogen bond	2.21	B:ASP437:OD2
Hydrophobic	1.60	E:DT8
Hydrophobic	4.26	B:ARG458
Hydrophobic	4.78	D:PHE1123
Hydrophobic	5.11	D:PHE1123
Hydrophobic	4.17	D:PHE1123
Hydrophobic	4.77	E:DT8
Hydrophobic	4.93	E:DT8
Hydrophobic	4.58	E:DT8
Hydrophobic	3.71	E:DT8
Hydrophobic	3.31	G:DG9
Hydrophobic	3.52	G:DG9
Hydrophobic	4.35	G:DG9
Hydrophobic	5.02	H:DA13
Hydrophobic	4.93	H:DA13
Hydrophobic	5.36	H:DA13
Hydrophobic	3.50	H:DA13
Hydrophobic	4.08	H:DA13
Hydrogen bond	2.21	B:ASP437:OD2
Hydrogen bond	2.21	B:ASP437:OD2

**Table 12:** Molecular docking analysis of compound 4 against the fungal enzyme lanosterol 14*α*-demethylase enzyme (PDB ID: 4wmz) on the basis of the type of bonds, bond distances, and interacting amino acids.

Bond type	Bond distance (Å)	Interacting amino acid of protein
Hydrophobic	5.43	A:ILE139
Hydrophobic	5.31	A:ILE139
Hydrophobic	4.67	A:LYS151
Hydrophobic	5.05	A:VAL154
Hydrophobic	4.99	A:VAL311
Hydrophobic	4.47	A:VAL311
Hydrophobic	5.46	A:ILE471
Hydrophobic	5.35	A:ILE471
Hydrophobic	3.57	A:VAL311
Hydrophobic	4.58	A:ILE139
Hydrophobic	4.62	A:LEU147
Hydrophobic	4.15	A:LYS151
Hydrophobic	4.93	A:LEU307
Hydrophobic	4.69	A:ILE139
Hydrophobic	4.68	A:VAL154
Hydrophobic	3.90	A:VAL311
Hydrophobic	3.97	A:LEU380
Hydrophobic	4.20	A:LEU380
Hydrophobic	5.21	A:LEU383
Hydrophobic	4.79	A:TYR126
Hydrophobic	5.32	A:PHE134
Hydrophobic	5.34	A:TYR140
Hydrophobic	5.20	A:PHE236
Hydrophobic	4.76	A:PHE236

## Data Availability

All the available data are incorporated in the manuscript and can be obtained from the research supervisor Dr. Ijaz Ahmad.
